The article "Segmentation and Classification of Heart Angiographic Images Using Machine Learning Techniques" was published in 2021. Journal: J Healthc Eng.

# Segmentation and Classification of Heart Angiographic Images Using Machine Learning Techniques

**DOI:** 10.1155/2021/6666458

**Published:** 2021-01-28

**Authors:** Abdullah, Muhammad Hameed Siddiqi, Yousef Salamah Alhwaiti, Ibrahim Alrashdi, Amjad Ali, Mohammad Faisal

**Affiliations:** ^1^Department of Computer and Software Technology, University of Swat, KPK, Mingora, Pakistan; ^2^Department of Computer Science, Jouf University, Sakakah, AlJouf, Saudi Arabia; ^3^Department of CS & IT, University of Malakand, Chakdara, KPK, Pakistan

## Abstract

Heart angiography is a test in which the concerned medical specialist identifies the abnormality in heart vessels. This type of diagnosis takes a lot of time by the concerned physician. In our proposed method, we segmented the interested regions of heart vessels and then classified. Segmentation and classification of heart angiography provides significant information for the physician as well as patient. Contradictorily, in the mention domain of heart angiography, the charge is prone to error, phase overwhelming, and thought-provoking task for the physician (heart specialist). An automatic segmentation and classification of heart blood vessels descriptions can improve the truthfulness and speed up the finding of heart illnesses. In this work, we recommend a computer-assisted conclusion arrangement for the localization of human heart blood vessels within heart angiographic imageries by using multiclass ensemble classification mechanism. In the proposed work, the heart blood vessels will be first segmented, and the various features according to accuracy have been extracted. Low-level features such as texture, statistical, and geometrical features were extracted in human heart blood vessels. At last, in the proposed framework, heart blood vessels have been categorized in their four respective classes including normal, block, narrow, and blood flow-reduced vessels. The proposed approach has achieved best result which provides very useful, easy, accurate, and time-saving environment to cardiologists for the diagnosis of heart-related diseases.

## 1. Introduction

Cardiovascular diseases caused first death many years ago in North America. Abnormality or blockage of coronary artery of the heart instigates it. In the last decade, very crucial developments were made to improve the diagnosis of patient in cardiology in order to increase the rate of survival. For the diagnosis of the coronary heart diseases, angiography is used.

There are four classes of the heart blood vessels, i.e., blood flow-reduced vessels, narrow vessels, block vessels, and normal vessels. It is very time-consuming and not so much significant to manually detect the classes of heart blood vessels in manual diagnoses. There are various artificial intelligence techniques and digital image processing modalities (computer-aided system) which efficiently segment and categorize the human heart blood vessels in angiography images [1]. The classification system in angiography obtains a sequence of images and chooses the section of interest (SOI) to segment an image, like left ventricle [2]. Intravenously sharpens improved heart angiogram X-ray was complete throughout a single inhalation clench, and echocardiograph-matching images were reconstructed with perception. Two investigators evaluated each part and section of the coronary artery greater than or equal to 3.0 millimeter having no stents and consociated them with algebraic average heart angiography. Patients were classified on the basis of average heart rate, and standard deviations are taken in three clusters [3]. To detect significant scratches of diameter greater than or equal to 50 percent decrease, diagnostic performance of data related to heart was contrasted with data of heart angiogram X-ray's quantification [4].

The article "Segmentation and Classification of Heart Angiographic Images Using Machine Learning Techniques" was published in 2021. Journal: J Healthc Eng.

Cardiology images are used a lot for analyzing and management of heart patients. A busy cardiologist is facing the increasingly unpromising task to keep informed of the current knowledge and the new changes in the analysis and treatment of diseases [5]. Techniques of imaginings, such as scoring of calcium in heart arteries and diagnosis of heart diseases with angiography, are achieved by revised dominion associated with present-day machine-learning approaches in the domain of heart diseases [6].

The framework will improve the clinical instruments and examination program in order to label and classify into images of the heart vessels of a human. When human heart vessels are classified and segmented automatically, it will help cardiologists to diagnose various heart infections. The goal of our research is to determine if the proposed image allotment methods are effective in classification and segmentation of human heart vessels. Our main attention is towards the classification of the human heart vessels in the field of practical cardiology. In various medical fields worked on, the main agony is the data which are not restful to relate to large quantities of models. The image information was taken from the research center of cardiology located in Hayatabad (HMC), Peshawar, Pakistan. There are 400 angiographic imaginings in the data set accumulated under the supervision of a heart doctor. These data consist of many conditions due to which human heart vessels are affected. For the purpose to help cardiologist in easily diagnosing various long-lasting heart diseases such as cardiac arrest, pain in the leg, and pain in the chest, the novelty of this propose work is that first time we categorize the ventricle heart vessels into four classes in supervision of a heart specialist/cardiologist. Furthermore, horizontal and vertical edge detection of heart vessels, which is explained in Segmentation, is new idea.

The article "Segmentation and Classification of Heart Angiographic Images Using Machine Learning Techniques" was published in 2021. Journal: J Healthc Eng.

## 2. Related Study

Langley et al. created an algorithm for myocardial ischemia classification. In this paper, the proposed method will improve the algorithm. The peak value of sensitivity of the Langley classifier is 99.0 percent. However, its lower specificity value is 93.3 percent. For the improvement of the specificity, this algorithm recategorizes the ischemic events of the Langley classifier. Support vector machine is used for classification. Standard deviation means, standard deviation peak value, and the starting standard deviation are the features used. The specificity is increased from 92.3 percent to 93.3 percent by the classifier. However, there is a disadvantage, i.e., the reduction in sensitivity from 99.0 percent to 97.5 percent as a result of which the total correctness is reduced from 95.6 to 94.8. The algorithm fulfills the promise of increasing the specificity. However, more work is to be done in order to find features that do not affect the sensitivity to decrease [7].

Automatic coronary artery centerline when extracted from 3D CT angiography (CTA) has significant clinical applications for diagnosing the atherosclerotic heart disease. Most of the work is dominated by segmentation where the complete coronary artery system is segmented like trees using a computer. However, the process, where various branches of vessels (defined by their medical semantics), is of much clinical significance and is performed manually. A hierarchical machine learning approach is proposed in this paper that will help in tackling of the tubular structure parsing problem in medical imaging. This framework will also help in parsing tasks of other tabular structures generically [8]. In this study, an intelligent system based on genetic-support vector machines is proposed. This intelligent system deals with the combination of feature extraction and classification from measured Doppler signal waveforms at the heart valve using the Doppler ultrasound. GSVM is used in this study for the diagnosis of heart valve diseases. The outcomes presented GSVM's success in detecting Doppler coronary sounds. The average rate of precise classifying rate was approximately 95 percent [9].

The categories of the infections in which coronary plaques play significant role to infect the heart with diseases were determined. Therefore, the previous focuses, either to detect specified class of coronary infections caused by plaque or to distinguish between infected and noninfected coronary vessels, ignore [10]. Various categories of coronial infections caused by plaque were detected or recognized using the data of affected patients. Typical imaging approaches such as electrocardiogram (ECG), computed tomography (CT), magnetic resonance imaging (MRI) and radiology tools of choice are used to diagnose cardiovascular diseases. All of these modalities will be impacted essentially and enduringly by machine level learning and neural network. However, the image processing context is discussed mainly with deep learning, and we present that the effect is more severe than this. Nonetheless, the procedure in which the outcomes brought to doctors are nontrivial, and we have also discussed our experience with this algorithm's deployment [11].

The article "Segmentation and Classification of Heart Angiographic Images Using Machine Learning Techniques" was published in 2021. Journal: J Healthc Eng.

With the beginning and speedy presentation of artificial intelligence (AI), Internet of things, mobile phones, and devices with sensors such as smart watch, we enter into the age of automated, isolated, and portable services. As directed by the World Health Organization (WHO), cardiovascular infection is the modern disease. However, prediction rate of coronary disease sufferers can be made conceivably and made excessive with initial finding and analysis. We portray a framework that observes robotized coronary heart health making full use of cell phone and wearable sensors [12]. The proposed technique is capable of reliably and efficiently assessing the position and radius of coronary vessels (arteries) in the heart, which is based on straight facts from the heart image data collection. The framework can be trained with minimal data on the train heart image and allows for rapid automated or interactive extraction of the coronary artery from CCTA heart images once trained [13]. The key aim of this work is to establish an automated method for CT images to detect calcified coronary plaques. In comparison to the avant-garde, both native and angio data sets are processed in this technique, and this dual information is used for identification and evaluation of calcified plaques. The success rate of the proposed method is stated by the authors as 85%. The research focuses only on the plaques being calcified [14]. The proposed method consists of preprocessing, extraction of features, and classification. Using preprocessing techniques, the vessels in the coronary image are enhanced, and then features are extracted from these images that are supplied to the CANFIS classifier. This classifier classifies the coronary image of the test given as either normal or abnormal. In addition, if the proposed method classifies the test image as irregular, the blockage is detected and segmented [15]. Coronary computed tomography angiography (CCTA) is now a well-established, noninvasive cardiovascular disease evaluation modality. The proposed framework is based on extracting data from CCTA as well as non-contrast-enhanced cardiac CT scans, and ML has been increasingly used to improve performance [16].

The article "Segmentation and Classification of Heart Angiographic Images Using Machine Learning Techniques" was published in 2021. Journal: J Healthc Eng.

## 3. Proposed Methodology

In the current era, numerous applications curiously want the high pixel quality in sense of resolving power to get improved images by means of low eminence info over separate apparatus such as angiography device angiogram, computer tomography scanner, and MRI. Medical imaging area investigation and finding are too much tough objectives to gain from very low-slung eminence images in sense of pixel quality and color scheme. On the basis of this thoughtful matter, the high resolving images are gained using the super resolution method with automated modalities. It is very thought-provoking objective to evaluate the imageries taken with angiogram equipment with low-slung pixel and color quality and composite tree-like arrangement as well as low accuracy and resolving power. Moreover, the classification and segmentation of human heart vessels also provides an appropriate background on the basis of images processing idea, and modalities can be very easily and flexibly evaluated. The proposed scheme consists of four key steps: adjustment of contrast, segmentation, features extraction and features selection, and classification with multiclass-assembled support vector machine. The proposed hierarchal method is used to achieve best result which provides very useful and time-saving environment for diagnosis of the heart-related diseases to the cardiologist/physician.

### 3.1. Contrast Adjustment

The first phase of the proposed method is contrast adjustment in which we increase the sharpness intensity of heart blood vessels which is obtained from angiography as shown in Figure 1.

### 3.2. Segmentation

In this phase, we divided the human heart angiographic image into *X*-axis and *Y*-axis edges as shown in Figure 2. After the division of vertical and horizontal edges, we combine both the edges to refine the shape of angiography images of tree-like structure. After the concatenation of vertical and horizontal edges, we apply Laplacian filter on the targeted image. Laplacian filter has two parameters: alpha and gamma which sort out the information below 0.5, respectively, on *X*-axis and *Y*-axis. Our proposed approach gives better results as shown in Figure 3.

### 3.3. Features Extraction and Selection

Here, in the proposed method, we extracted the local binary pattern (LBP) and histogram-oriented gradient (HOG). In LBP, we take a mask which is further used on a target image and take binary patterns, while in HOG, we divide the image into subsections, take histogram of every section, and then combine the section histogram. When we extracted both LBP and HOG features, we combined both the features and saved it in feature vector for classification. Examples of LBP features, pixel value of image, and selected mask are given in Tables 1 and 2, respectively.

The article "Segmentation and Classification of Heart Angiographic Images Using Machine Learning Techniques" was published in 2021. Journal: J Healthc Eng.

### 3.4. Classification

The final step is classification when we extract features from LBP and HOG and then combine it and save it in a feature vector. On the basis of these features, we trained a multiclass-assembled classifier as support vector machine on the basis of cardiovascular images data from angiogram images. Here, in the proposed method, we select a vector which best fits the data after extraction of features from the proposed data set according to the selected framework. So, for this purpose, we select a method called principle component analysis with the help of which we reduced the redundant features. The cross validation used here is as follows: 30% data used for testing purpose and 70% for training purpose in the data set. The proposed framework for classification and segmentation of heart images is shown in Figure 4.

## 4. Results and Discussion

Investigation remained accepted and appropriate on the basis of human heart angiography blood carrier's data collected from two hospitals of Peshawar cardiology center of complex hospital Hayatabad and teaching hospital Khyber Peshawar. The proposed system is simulated on the MATLAB tool. It is a well-established tool used by researchers for statistical and data analysis due to diverse set of libraries and gives optimized, efficient, and accurate results. To collect the minced multiplicity of human heart blood carriers, heart specialists were desired to classify the human heart angiographic imageries into their consistent categories, i.e., normal blood carrier, blood flow-reduced carrier, block blood carrier, and narrow blood carrier. Segmentation and classification are applicable for ventricular vessels, which may be normal vessels, block vessels, blood flow-reduced vessels, and narrow vessels. The solid results were predictable to the database and are accumulated to judge the result of various catalogue procedures. The investigation was accomplished on 400 data sets of human heart blood carrier images, consisting of both defective and nondefective images of human heart vessels. From acknowledged facts storehouse of descriptions, only the heart angiography images were integrated and catalogued into their own 4 categories as shown in Figure 5. The consequences after that accompanying with the pulverized fact to evaluation the suitability of the predicted heart angiography classification technique. The essentials in between examinations are clarified in the succeeding scraps.

The article "Segmentation and Classification of Heart Angiographic Images Using Machine Learning Techniques" was published in 2021. Journal: J Healthc Eng.

The data set after findings containing four-hundred images were collected from two hospitals of Peshawar in which one is the center of heart diseases cardiac research center of Hayatabad and other one is the teaching hospital of Khyber. All data set samples were in Joint Photographic Experts Group with dimension according to the coordinate system *X*-axis 960 while *Y*-axis is 1080 per pixel. Due to the requirement of MATLAB, the data set was adjusted to 128 by 128. Details of the data with repository are given in Table 3.

The convinced evaluation was accomplished to check the classification consequences of the proposed method. In the proposed method, six cardiologists were involved during independent evaluation to point out the parts of human heart in images; these image data sets of different patients are taken through a device called angiogram, and the process is called angiography. Under the supervision of a cardiologist, respective categories, i.e., normal, blood flow-reduced, narrow, and block vessels were set physically. The region of interest (segmentation) by physically of human heart angiography data set as booked minced truth for valuation with heart vessels segmentation by suggested framework. There are three metrics used to find out the false-positive ratio, false-negative ratio, and *F*-measure as follows:

False-positive ratio = FP/TN + FP.

False-negative ratio = FN/TP + FN.

*F*-measure = FPR + FNR/FPR + FNR^∗^2.

Here, TP is true positive, FP is false positive, and FN is false negative. True positive specifies the interest pixel, true negative specifies noninterested value, false positive identifies the heart vessel's nonconcerned section, and false negative identifies the section where, in the suggested procedure, we are not intended in the heart vessel pixel. Wrongly accepted as noninteresting cell pixels show that the *F*-measurement of the modalities for four-hundred blood vessels in the heart vessels in all kinds of images in both parts of perception and in the dissecting of vessels in machine learning sections is more than 85 percent. This particular consequence of dissection is more important, widespread, careful, and far closer to the manual splitting off of heart angiography, i.e., real evidence. The false positive, false negative, and *F*-measure results are shown in Figure 6 and Table 4 [18].

The article "Segmentation and Classification of Heart Angiographic Images Using Machine Learning Techniques" was published in 2021. Journal: J Healthc Eng.

In pattern recognition, information retrieval, and classification (machine learning) precision (also called positive predictive value) is a fraction of the relevant instances among the retrieved instances, while retrieval (also known as sensitivity) is a fraction of the retrieved relevant instances among all relevant instances. Statistical approaches for the study of data from radioimmunoassay are provided. The viability of using the logic transformation has been empirically checked, and the benefits arising from the study of the data in this manner are considered. The statistical transformations take into account the heteroscedasticity of the error inherent in a heart angiography normal and the abnormal extant in the confidence intervals about the estimates of the values of individual samples [14].

The specificity = TN/(TN + FP), precision = TP/(TP + FP), and the results are shown in Figures 7 and 8, respectively.

The accuracy of each class is shown in Figure 9 and is given as follows: accuracy = number of correct prediction/total number of prediction.

The accuracy of the overall frame framework is shown in Figure 10 and is given as follows: accuracy = one prediction/total number of prediction.

## 5. Conclusion

The suggested method of segmentation is to concatenate the identification of the edge and the Laplacian filter. In the proposed method, the combined edge detection system and the Laplacian filter provide full information from cardiac angiographic images. Edge detection plays an important role in the tree, such as the structure of cardiac angiographic images, and the Laplacian filter has two alpha and beta parameters that extract information from cardiac angiographic images below 0.4 on both coordinates. In this paper, we first segment the input image and extract function that gives the best accuracy to the multi-SVM Classifier. The method, however, suffers from the complete classification of narrow boats, but the overall result of the proposed modality is good enough. Efficiency is improved due to the execution of each stage of the framework precisely and mostly in the resizing of images to save processing time. The proposed method provides the doctor/cardiologist and patient with a simple and reliable, time-saving diagnostic approach, as well as a health-related approach [19–21].

## Figures and Tables

**Figure 1:** Divergence balance.

**Figure 2:** The process of segmentation.

**Figure 3:** Segmentation approaches [17] with the proposed system.

**Figure 4:** The proposed framework for classification and segmentation of heart images.

**Figure 5:** Results after classification. (a) Block vessels. (b) Normal vessels. (c) Blood flow-reduced vessels. (d) Narrow vessels.

The article "Segmentation and Classification of Heart Angiographic Images Using Machine Learning Techniques" was published in 2021. Journal: J Healthc Eng.

**Figure 6:** Results of false positive, false negative, and *F*-measure from the data set.

**Figure 7:** Specificity.

**Figure 8:** Precision.

**Figure 9:** Accuracy.

**Figure 10:** Performance of the entire framework.

**Table 1:** Pixel value of an image.

55	66	45

77	60	32

52	33	88

**Table 2:** Pattern after applying mask which is 0100110001.

0	1	0

1	0	0

0	0	1

**Table 3:** Classes with number of images.

S. No.	Human heart interior groups	Number of data sets
I	Block	Hundred
II	Narrow	Hundred
III	Reduction of blood flow	Hundred
IV	Normal	Hundred
V	Overall	Four-hundred

**Table 4:** Overall accuracy of the proposed system.

Heart angio image types	False positive	False positive	*F*-measure
Normal vessels	0.002	0.095	0.882
Block vessels	0.003	0.045	0.971
Blood flow-reduced vessels	0.000	0.109	0.963
Narrow vessels	0.122	0.097	0.882

## Data Availability

The data used to support the findings of this study are included within the article.
